The article "H2S attenuates endoplasmic reticulum stress in hypoxia-induced pulmonary artery hypertension" was published in 2019. Journal: Biosci Rep.

# H_2_S attenuates endoplasmic reticulum stress in hypoxia-induced pulmonary artery hypertension

**DOI:** 10.1042/BSR20190304

**Published:** 2019-07-08

**Authors:** Jianjun Wu, Weili Pan, Chao Wang, Hui Dong, Lei Xing, Jingbo Hou, Shaohong Fang, Hulun Li, Fan Yang, Bo Yu

**Affiliations:** 1 Department of Cardiology, The Second Affiliated Hospital of Harbin Medical University, Harbin, Province Heilongjiang, China; 2 The Key Laboratory of Myocardial Ischemia, Chinese Ministry of Education, Harbin, Province Heilongjiang, China

**Keywords:** ER stress, Hydrogen sulfide, Nox-4, Pulmonary arterial hypertension, pulmonary artery smooth muscle cells

## Abstract

**Background:** Previous studies have found that hydrogen sulfide (H_2_S) has multiple functions such as anti-inflammatory, antioxidative in addition to biological effects among the various organs. Exaggerated proliferation and resistance to apoptosis of pulmonary artery smooth muscle cells (PASMCs) is a key component of vascular remodeling. We hypothesized that endogenous bioactive molecular known to suppress endoplasmic reticulum (ER) stress signaling, like H_2_S, will inhibit the disruption of the ER-mitochondrial unit and prevent/reverse pulmonary arterial hypertension (PAH).

** Methods and results:** A hypoxic model was established with PASMCs to investigate the possible role of H_2_S in PAH. Effects of H_2_S on proliferation of PASMCs were evaluated by CCK-8 and EdU assay treated with or without GYY4137 (donor of H_2_S). H_2_S significantly inhibited hypoxia-induced increase in PASMCs proliferation in a dose-dependent manner. H_2_S by intraperitoneal injection with rats both prevented and reversed chronic hypoxia-induced pulmonary hypertension in rats, decreasing pulmonary vascular resistance, pulmonary artery remodeling and right ventricular hypertrophy, and improving functional capacity without affecting systemic hemodynamic. Exogenous H_2_S suppressed ER stress indexes *in vivo* and *in vitro*, decreased activating transcription factor 6 activation, and inhibited the hypoxia-induced decrease in mitochondrial calcium and mitochondrial function.

**Conclusion:** H_2_S effectively inhibits hypoxia-induced increase in cell proliferation, migration, and oxidative stress in PASMCs, and NOX-4 might be the underlying mechanism of PAH. Attenuating ER stress with exogenous H_2_S may be a novel therapeutic strategy in pulmonary hypertension with high translational potential.

## Introduction

Pulmonary arterial hypertension (PAH) is a complex disease characterized by a progressive narrowing of the distal pulmonary arteries [1], which causes right ventricular failure and death. Excessive proliferation and impaired apoptosis of pulmonary artery smooth muscle cells (PASMCs) contribute to vascular obstruction in patients with PAH [2,3]. These pathological structural abnormalities due to vasoconstriction and vascular remodeling are accompanied by marked and sustained elevation of pulmonary vascular resistance. Hypoxia is found to be crucial in the development of PAH. Recent studies have demonstrated that inflammatory responses also may cause lung damage and PASMCs fibrosis, leading to progressive impairment of lung function [4,5].

Reactive oxygen species (ROS) have been shown to play a key role in promoting abnormal function in pulmonary arterial smooth muscle and endothelial cells in PAH [6,7]. Nicotinamide adenine dinucleotide phosphate (NADPH) oxidase (Nox4)-derived ROS and endoplasmic reticulum (ER) stress have been implicated in the vasculature Nox4, an ER resident capable of producing ROS, acts as a proximal signaling intermediate to transduce ER stress-related conditions to the unfolded protein response, a homeostatic corrective mechanism [8].

Hydrogen sulfide (H_2_S) has emerged as an important member of the family of gas transmitters, which also include nitric oxide and carbon monoxide. The physiological and pathophysiological roles of H_2_S in the regulation of cardiovascular function, such as modulated metabolic state, mitochondrial function, cellular redox status, and cell apoptosis, have received more attention [9,10]. Our previous studies demonstrated that H_2_S exerts its protective effects on myocardial injury through the amelioration of mitochondrial function [11]. However, the detailed mechanism underlying the protective effects of H_2_S against PAH is not fully understood. Despite major advances in the field, current therapies for PAH remain poorly effective in reversing the processing or significantly improving long-term survival. Accordingly, the present study aimed to analyze the H_2_S regulation of ER stress and the role of H_2_S/Nox4 in the pathogenesis of PAH in rats.

## Materials and methods

### Animals

The present study was approved by the Institutional Experimental Animal Care and Ethics Committee of Harbin Medical University (Heilongjiang, China). All animal care and experimental protocols complied with the Animal Management Rules of the Ministry of Health of the People’s Republic of China (documentation number 19890503) and the Guide for the Care and Use of Laboratory Animals of Harbin Medical University (Heilongjiang, China). The present study included 40 male Sprague–Dawley rats, weighing 250–280 g, which were obtained from the Experimental Animal Centre, Harbin Medical University (Heilongjiang, China) and kept in our laboratory animal husbandry facility until the experiments. Rats were acclimated for 1 week before experiments, with unrestricted access to demonized water and standard rat chow with no other restrictions. Before and throughout the study, rats were kept at room temperature (22°C) at 30–70% humidity on a 12-h day/night cycle with the lights turned on at 7:00 a.m. No deaths occurred before intervention.

### Materials

GYY4137 (GYY) (SML0100) and thiazolyl blue tetrazolium bromide (M2128) were both purchased from Sigma Chemical (St. Louis, MO). GYY4137 is one kind of H_2_S donor. DMEM/F12 (SH30023.01) and fetal bovine serum (FBS) were purchased from HyClone. 2′,7′-dichlorofluorescein diacetate (DCFH-DA) was obtained from Beyotime (Shanghai, China). N-acetyl-l-cysteine (NAC), siRNA Nox4 were purchased from Cell Signaling Technology (Beverly, MA). Lipofectamine 2000 and ER-tracker were both obtained from Invitrogen (Carlsbad, CA). Primary antibodies are provided by Cell Signaling Technology (Beverly, MA, U.S.A.).

### MTT assay

PASMCs (5 × 10^3^ cells/well) were seeded in 96-well plates and treated with 0.4 mg/ml MTT diluted in low glucose FBS-supplemented complete medium for 4 h at 37 °C. After treatment, medium was removed and plates were left to air-dry overnight. Formazan crystals were resuspended in DMSO and absorbance was measured at 560 nm with background at 670 nm on a Cytation 5 plate reader.

### Echocardiography and hemodynamics

Cardiac output (CO) was assessed on isoflurane-anesthetized animals by echocardiography using the Vevo770 imaging system with the 707B (30 MHz) and 716 (15 MHz) probes for rats. The CO was calculated after determining the left ventricular outflow tract diameter (LVOT), aortic velocity-time integral (AoVTI), and heart rate (HR) with the following formula:

$$\text{CO }=\;7.85*{\text{LVOT}}^{2}*\text{AoVTI}*\text{HR}/1000$$

Pulmonary artery acceleration time was measured by echocardiography as previously described [12]. Total pulmonary resistance was calculated by the ratio of mean pulmonary arterial pressure to CO. Pressures from the right atrium, right ventricle, and pulmonary arteries were recorded continuously, and mean pulmonary artery pressure was calculated electronically (Power Laboratory, with Chart software 5.4, ADInstruments).

### Treadmill test

Animals were placed on a calibrated, motor-driven treadmill (Treadmill Simplex II, Columbus Instruments) and run once a week (three times total) on an undemanding protocol to allow familiarization with the test. Afterward, animals from each therapy group were run until failure with the following protocol: 3 min at 10 m/min, 3 min at 12 m/min, 20 min at 14 m/min, 20 min at 16 m/min, and 18 m/min until failure. Failure was defned as greater than five consecutive seconds on the shocker grid, and the test was terminated.

### Observation of intracellular ROS content

Intracellular ROS was determined by the oxidative conversion of cell permeable DCFH-DA to fluorescent 2′,7′-dichlorofluorescein (DCF). At the end of the indicated treatments, the HPASMCs were washed and incubated with 10 μmol/l DCFH-DA solution at 37°C for 20 min in darkness. Intercellular DCF fluorescence was observed over the entire field of vision using a fluorescence microscope connected to an imaging system (BX50-FLA; Olympus, Tokyo, Japan). The mean fluorescence intensity (MFI) of DCF from four random fields was analyzed using ImagePro Plus software (version 6.0, Media Cybernetics).

### Measurement of superoxide dismutase and catalase activities

The activities of superoxide dismutase (SOD) and catalase (CAT) were determined by a Total Superoxide Dismutase Assay Kit with NBT (Beyotime Biotechnology, Shanghai, China) and a Catalase Assay Kit (Beyotime Biotechnology, Shanghai, China) following the manufacturer’s instructions as previous reports [13]. The activity results were expressed as U/mg protein.

### Determination of malondialdehyde

The levels of malondialdehyde (MDA) were measured using commercial assay kits (Beyotime Biotechnology, Shanghai, China) according to the instructions provided by the manufacturer as previously described [14].

### Determination of MPTP opening

Calcein-AM is a non-fluorescent, cell permeable, and hydrophilic compound that is widely used for detection of cell viability. In live cells, the hydrolysis of calcein-AM by intracellular esterase produces strongly green fluorescent calcein, a hydrophilic compound that is well retained in the cell cytoplasm. Shortly, cardiac cells were incubated for 20 min with the fluorescence dye, calcein-AM (1 μM), which accumulates in cytosolic compartments, including the mitochondria. Then the medium was changed to calcein-free medium containing 1 μM CoCl_2_ and incubated at 37 °C for 20 min in the dark. The fluorescence from cytosolic calcein was quenched by the addition of CoCl_2_, (1 mM) for 20 min, while that from the mitochondrial calcein was maintained. MPTP opening was induced by adding ionomycin (5 μM). Then the cells were washed with ice-cold PBS (pH 7.2) for four times and the fluorescence intensity of cells exposed to high glucose or untreated control cells was measured with excitation at 490 nm and emission at 520 nm. The percentage loss of calcein fluorescence was used to determine MPTP opening.

### Caspase activity assays

Caspase activity assays in multi-well plate formats represent powerful tools for understanding experimental modulation of the apoptotic response. Caspase 3, Caspase 8 and Caspase 9 Multiplex Activity Assay Kit (Fluorometric) (ab219915) are purchased by Abcam. It a fluorescent assay that detects the activity of caspase-3/-8/-9 in cell lysates. We followed the protocol in https://www.abcam.com/ps/products/219/ab219915/documents/. Subtract blank readings from all measurements (control and treated)—using fluorescent intensity, determine fold change between control and treated cells. The fluorescence intensity was measured with FlexStation fluorescence microplate reader at the indicated wavelength. Caspase 3 (Ex/Em = 535/620 nm), Caspase-8 (Ex/Em = 490/525 nm), and caspase-9 (Ex/Em = 370/450 nm), activities can be detected in a single assay without interferences from other caspases.

### Statistical analysis

All values were given as the means ± the standard error of the mean (S.E.M.) for at least three independent experiments’ replicates. Statistical analysis was analyzed with Newman *t* test or ANOVA as appropriate using GraphPad Prism 7 for Windows platform (GraphPad Software, San Diego, CA). *P*<0.05 was considered statistically significant.

## Results

### Exogenous H_2_S inhibits hypoxia-induced PASMCs proliferation

GYY4137 has been well-known as a novel H_2_S donor with its vasodilatory and antihypertensive activities [15]. Since neointimal hyperplasia results from the abnormal proliferation and migration of PASMCs, therefore, we first evaluated the effect of GYY4137 on PASMCs viability. Using the MTT assay to measure metabolic activity following treatment, we identified 109 ± 4 μM as the EC_50_ for GYY4137 in PASMCs (Figure 1A). Flow cytometry analysis determined that the total viable cell number following GYY4137 treatment was reduced in a dose-dependent manner. Treatment with 100 μM GYY4137 significantly reduced the total viable cell number (*P*<0.05, Figure 1B) without increasing the total number of dead cells (*P*=NS compared with control, Figure 1C). Treatment with 320 μM GYY4137, however, did increase cell death suggesting high-dose GYY4137 toxicity (*P*<0.05, Figure 1C). Next, apoptosis analysis was performed to investigate if the observed reduction in viable cell number was through GYY4137-induced PASMCs apoptosis. Flow cytometry results showed that 50 and 100 μM GYY4137 treatment did not increase either the total apoptotic cell population or the proportion of early apoptotic, late apoptotic, or dead cell subpopulations within the apoptotic cell population (*P*=NS, Figure 1D). Taken together, our results suggested that 100 μM GYY4137 reduced PASMCs total cell number by inhibiting cell proliferation, while cell apoptosis contributed more to the reduction in total PASMCs number only at toxic GYY4137 concentrations (>200 μM ).

**Figure 1:** The 100 µM GYY4137 reduced PASMCs number without inducing apoptosis PASMCs in 25 mM glucose were synchronized overnight and then stimulated with different concentrations of CA. (**A**) Metabolic activity analyzed by MTT of PASMCs treated with GYY4137 dose range (EC_50_ = 109 ± 4 μM) (*n*=4 independent experiments with eight replicates). (**B**) Quantitation of total viable PASMCs after treatment with increasing doses of GYY4137. (**C**) Quantitation of total dead PASMCs after GYY4137 treatment. (**D**) Quantitation of early apoptotic, late apoptotic, and dead PASMCs after treatment with increasing doses of GYY4137. Significant increase shown is only in the late apoptotic cell population. No significant change in other subpopulations. (B–D) *P<0.05 compared with control (0 µM GYY4137); data presented as means ± SEM (*n*=3 independent experiments in triplicate).

### Exogenous H_2_S reversed hypoxia-induced proliferation, migration of PASMCs

Increased cell proliferation of PASMCs induced by hypoxia is a key feature in PAH, thus we investigated the effect on PASMCs proliferation in hypoxia cell model. CCK-8 assay and EDU assay were used to evaluate the level of PASMCs proliferation treated with 0 (vehicle), 100 μM GYY4137. As shown in Figure 2A, PASMCs cultured under hypoxia condition showed a significantly increased proliferation, while 100 μM GYY4137 could significantly inhibit hypoxia-induced PASMCs proliferation. EDU assay also revealed a significant anti-cell proliferative effect of GYY4137 in hypoxic PASMCs (Figure 2B). The 100 μM GYY4137 showed comparable inhibition effects on PASMCs proliferation cultured under hypoxia in CCK-8 assay, thus we used 100 μM GYY4137 in subsequent experiments.

**Figure 2:** GYY4137 reverses hypoxia induced dysfunction in cell proliferation, cell migration, generation of ROS in PASMCs (**A**) Increased OD450 value in CCK-8 assay of PASMCs with hypoxia compared with cells cultured under standard condition, and ((**B**) Scale bars, 100 μm) representative images of EdU assay. PASMCs under hypoxia showed significant narrow width of scratch in scratch test assay ((**C,D**), Scale bars, 100 μm), increased cell number in lower chamber in Transwell assay (**E,F**, original magnification ×200), and ROS generation (**G,H**, original magnification ×200), while treatment of DHA inhibited hypoxia-induced increase in cell migration. The data are presented as the mean ± standard error of mean (S.E.M), one-way ANOVA, followed by Tukey’s post-hoc test; *P<0.05, vs normoxia group; ^#^*P*<0.05, vs hypoxia group.

Increasing migration of smooth muscle cells contribute to the development of PAH, thus we investigated the effect of GYY4137 on PASMCs migration in hypoxia cell model by scratch test assay and transwell assay. PASMCs cultured under hypoxia condition showed wider scratch than cells treated with 100 μM GYY4137 for 24 h (Figure 2C,D). As shown in Figure 2E,F, PASMCs migration was significantly enhanced in chronic hypoxia, while cell migration was obviously reversed by GYY4137 treatment. Our results also showed that generation of ROS was decreased in GYY4137 group compared with hypoxia group (Figure 2G,H).

### Exogenous H_2_S prevented and reversed pulmonary hypertension in rats and down-regulated ER-related proteins’ expressions in PAH rats

To verify whether exogenous H_2_S could be a potential PAH therapy, we used Wistar rats exposed to 4 weeks of chronic hypoxia (Hypoxia) treated with GYY4137 in a prevention (intraperitoneal injection with GYY4137 starting at the day of chronic hypoxia exposure and continuing for 4 weeks). Rats treated with GYY4137 had lower mean pulmonary artery pressure and total pulmonary resistance compared with hypoxia group (Figure 3A,B).

**Figure 3:** GYY4137 prevents chronic hypoxia-induced PAH (**A**–**D**) Chronic hypoxic rats treated with GYY4137 had lower mean pulmonary artery pressure (mPAP; top left), total pulmonary resistance (bottom left), decreased right ventricle/left ventricle (RV/LV)+septum (top right), and improved treadmill running distance (bottom right) compared with vehicle-treated rats (*n*=9–15 rats per group; *P<0.05 vs normoxic vehicle; #*P*<0.05 vs hypoxic vehicle; red lines represent mean values). GYY4137 had no significant effects on normoxic rats. Each point represents one animal. (**E**) GYY4137 reduces the percent medial wall thickness (%MWT) in the resistance PAs (50- to 100-μm diameter) in the chronic hypoxic models of PHT. Images show Hematoxylin and Eosin-stained resistance PAs from vehicle- and GYY4137-treated animals (*n*≈15 vessels per animal, five animals per group; *P*<0.05), Scale bars, 50 μm. (**F,G**) GYY4137 reduces ER stress-related proteins in PAH model. H_2_S in prevention and reversal protocols reduces ATF6/ GRP78/caspase-12 and p-PERK protein expressions in hypoxia–PAH rats (mean data obtained from blot of *n*=5 rats per group; *P<0.05 vs normoxic vehicle; ^#^*P*<0.05 vs hypoxic vehicle). The upper trace of each group shows representative blots of the respective proteins, and the lower panels show the bar graphs summarizing the immunoblot data.

Similar to the vehicle group, GYY4137 group had decreased total pulmonary resistance (Figure 3C). Meanwhile, treadmill test revealed that decreased afterload resulted in lower right ventricular hypertrophy as well as improved functional capacity (Figure 3D).

Consistent with the improved hemodynamics, GYY4137-treated PAH animals had reduced medial wall thickening (MWT) of the resistance PAs (50- to 100-μm diameter) and reduced muscularization (in >50-μm-diameter PAs) (Figure 3E).

The expression of ER stress-associated proteins was analyzed by Western blotting to elucidate whether the cytoprotective effect of H_2_S reduced ER stress against hypoxia-induced injury. The expression of GRP78 and p60 ATF-6 in pulmonary artery tissues increased in PAH groups compared with control (*P*<0.05). The expression of GRP78 and ATF-6 decreased significantly in the PAH+GYY4137 groups compared with the PAH groups (*P*<0.05) (Figure 3F). The expression of p-PERK increased significantly in PAH groups compared with control rats (*P*<0.05), and exogenous H_2_S treatment decreased their expressions (*P*<0.05) (Figure 3G).

### Exogenous H_2_S inhibit in oxidative stress and mitochondrial calcium in hypoxia-induced PASMCs

Evidence has demonstrated that H_2_S can suppress ROS production as an ROS scavenger and increase SOD activity in various cells. Our team has reported that H_2_S is capable of suppressing ROS production and that ROS scavengers inhibit both apoptosis and autophagy [16]. Thus, we hypothesized that exogenous H_2_S protected function through inhibiting ROS production. Our results showed that both total (Figure 2G) and mitochondrial ROS production were significantly increased in the hypoxia group whereas these changes were suppressed by GYY4137 treatment (Figure 4A). To test how exogenous H_2_S suppressed ROS production, we examined SOD (Mn-SOD) and CAT (mito-CAT) activity in PASMCs mitochondria. Our data revealed that hypoxia impaired Mn-SOD and mito-CAT activity and this alteration was attenuated by GYY4137 treatment (Figure 4B). Our results indicated that exogenous H_2_S markedly increased mitochondrial Mn-SOD and mito-CAT activity, which showed that exogenous H_2_S could suppress mitochondrial ROS production a step further.

**Figure 4:** GYY4137 inhibits oxidative stress and mitochondrial calcium in hypoxia-induced PASMCs (**A**) Effects of GYY4137 on hypoxia-induced overproduction of ROS in mitochondria of PASMCs. Random micrographs of mitosox-derived fluorescence in PASMCs. Quantitative analysis of the MFI was obtained in the indicated groups. Data are the means ± SEM (*n*=3). *P<0.05 compared with normoxia, #*P*<0.05 compared with hypoxia. Original magnification ×200. (**B**) Effects of GYY4137 on SOD, CAT, and MDA activity in PASMCs. Data are the means ± SEM (*n*=3). *P<0.05 compared with normoxia, #*P*<0.05 compared with hypoxia. (**C**) Imaging of mitochondrial permeability transition pore (mPTP) opening with calcein. PASMCs were treated with: normoxic, hypoxia, hypoxia+GYY4137 (100 µM), hypoxia+NAC, and then further incubated for 48 h. The MPTP opening was measured by staining with calcein-AM and COCl_2_ (*n*=5 independent preparations). (**D**) Caspase activity of -3, -8, and -9 in PASMCs. The results were expressed as the mean ± S.E.M. (*P<0.05 vs hypoxia group, *n*=3).

To examine whether calcium-dependent apoptosis induced by ER stress is mediated through MPTP, we stained PASMCs for calcein/Co^2+^ to test opening of MPTP. We found the mitochondrial calcein in the cytoplasm decreased gradually after hypoxia treatment. Treatment with GYY4137 significantly inhibited MPTP opening at 48 h after hypoxia while treatment with NAC did not (Figure 4C).

In order to demonstrate the anti-apoptotic effect of GYY4137 in hypoxia-induced PASMCs, we examined the activity of caspase-3, -8, -9. In hypoxic group, caspase activity is significantly increased, compared with control group. Whereas, treatment with GYY4137 decreased caspase activity (Figure 4D).

### GYY4137 inhibits Nox4 expression in ER

To better characterize exogenous H_2_S affection on redox signaling in PASMCs and to evaluate whether Nox/ROS regulation is compartment specific and differentially regulated in PAH, we investigated the subcellular localization of Nox4. Expression of Nox4 was assessed by immunoblotting after cell fractionation (Figure 5) in plasma membrane, nuclear/ER fraction, and isolated ER in both strains. Housekeeping protein used for cell membrane was Na/K ATPase, for ER was calreticulin, and histone deacetylase 3 (HDAC3) for the nuclear/ER fraction. Nox4 levels were detected in all fractions. Our results show that Nox4 were significantly increased in the ER of PASMCs from PAH rats (Figure 5A), treatment with GYY4137 decreased the expression of Nox4 in all fractions. Our findings indicate that H_2_S decreases the expression of Nox4 via subcellular compartments, particularly ER and nucleus. The ER is a site of protein synthesis and a platform of stress signaling pathways that may be particularly important in oxidative stress in PAH and was further investigated in our studies.

**Figure 5:** GYY4137 inhibits hypoxia-induced ER stress via Nox4 Subcellular localization of Nox4 in PASMCs from control and hypoxia-induced PAH rats (PAH). Expression of Nox4 in isolated plasma membrane, nuclear fraction, and isolated ER (**A**). Results are expressed as mean ± SEM of three separate experiments and were normalized by Na/K ATPase (plasma membrane marker), HDAC3 (nuclear marker), or calreticulin (ER marker). *P<0.05 vs control rats. Nox4 siRNA was used to decrease Nox4 expression in control and hypoxia group of PASMCs. ER stress was assessed by the expression of CHOP (**B**) and ER tracker staining (**C**) in cells transfected with Nox4 siRNA (50 nM). Original magnification ×400. Results are expressed as mean ± S.E.M. of three separate experiments. *P<0.05 vs hypoxia+CtlsiRNA; ^#^*P*<0.05 vs hypoxia group.

PASMCs were cultured with hypoxia and GYY4137 to induce ER stress to demonstrate a link between ER stress and the expression of proteins involved in ROS activation. NOX4 expression levels were higher in the hypoxia-cultured group than those in the GYY4137 treatment group. The scrambled peptide control for Nox4 had no effect on ROS generation or ER stress-related protein, CHOP. In addition, Nox4 with short interfering RNA and treatment with GYY4137 both down-regulated basal ROS levels in PASMCs as determined using quantitative Western blotting (Figure 5B). We determined whether Nox4 was necessary for increased ROS-induced cell ER stress in the presence of hypoxia using siRNA-mediated silencing of Nox4 in PASMCs. Notably, GYY4137 treatment and transfection with Nox4 siRNA fully protected PASMCs against hypoxia-induced ER stress, as measured by ER-tracker (Figure 5C). These findings suggest that Nox4 and GYY4137 are constitutively active in resting conditions and are responsible for decreased basal ROS generation and ER stress in PASMCs in PAH rats.

## Discussion

PAH is a type of pulmonary hypertension that primarily affects the pulmonary vasculature. But the pathogenesis of hypoxic pulmonary hypertension has not been fully understood yet. Overproduction of ROS can result in the progression of pulmonary vascular remodeling [17–19]. H_2_S is an essential small molecule in human physiology. Although quite toxic, H_2_S is produced endogenously and performs important regulatory functions in the cardiovascular, immune, nervous, and respiratory systems [20,21]. Varied interactions with intracellular thiols, reactive oxidants, and protein transition-metal centers are highly dynamic and sensitive to fluctuations in redox homeostasis. Furthermore, H_2_S is implicated in a number of diseases such as cancer, neurodegeneration, and heart disease. Hence, exogenously delivered H_2_S as a therapeutic agent is an active area of intrigue and research [22,23]. Our previous work revealed that the endogenous CSE/H_2_S pathway was down-regulated in STZ-induced diabetes cardiomyopathy [11], meanwhile, H_2_S also could exert antioxidant effects *in vivo* and *in vitro* [24]. ROS and NO was reported to contribute to the pathophysiology of hypoxia-mediated PAH. Based on these sutdies, we hypothesized that H_2_S might act as an antioxidant in PAH and protect the body from oxidative injury. A cellular signaling pathway linked to apoptosis, fibrosis, and contractility is ER stress [12]. The lumen of the ER, which is vital in maintaining low cytosolic Ca^2+^ levels, contains a multitude of calcium-binding chaperone proteins responsible for protein folding. A disruption in ER folding capacity, which can occur following a variety of cellular stresses (oxidative, inflammatory, and energy/calcium depletion), leads to the misfolding and aggregation of proteins within the ER lumen: a process known as ER stress. Following ER stress there is an initiation of the unfolded protein response (UPR), a complex signaling network, which acts in the short term to restore ER homeostasis [25,26].

In human vasculature, there are mainly four isoforms NOX1, NOX2, NOX4, and NOX5. The activation mechanism of NOX4 is not fully understood. Tejero et al. [27] indicates that sequence between helics V and VI of NOX4 seems to provide steric hindrance to show down superoxide release. Previously we found that hypoxia increased mitochondrial superoxide via specific activation of NOX4 in PASMCs. Moreover, we demonstrated that these effects are accompanied by an increase in Nox4 and TGF, proteins suggesting that mitochondrial NOX4 represents a major source of oxidative stress that may subsequently cause functional damage of cells [28]. A corresponding study found that mice deficient in NOX4, but not NOX1, are protected from hypertension [29].

We hypothesize that the potential of exogenous H_2_S to decrease ROS-mediated PASMCs apoptosis through the SR and mitochondria subjected to hypoxia. Nox4-derived ROS contributes to oxidative and ER stress through oxidation of proteins that influence vascular function in pulmonary hypertension. To address this, we examined in PASMCs the subcellular compartmentalization and ROS-generating function of NOX4 and investigated how oxidative stress impacts the oxidative proteome focusing on reversible and irreversible oxido-reductive modifications and explored the role of ER stress in these processes [30].

In our study, we demonstrated that GYY4137 treatment reduced proliferation and induced apoptosis, *in vivo* and *in vitro*, reversing and preventing the pulmonary vascular remodeling of PAH (Figure 2). Increased cytosolic calcium ([Ca^2+^]cyt), which is regulated by inhibition of H_2_S generation that controls calcium influx, as well as Ca^2+^ sequestration within the ER and mitochondria, contributes to the contractile, hyperproliferative, and anti-apoptotic phenotype of PASMCs.

Depending on the degree and duration of ER stress in specific cell types, the mechanism between pro-apoptosis and pro-survival ER stress pathway is complex. ER stress was a potential candidate as it had been implicated in death receptor signaling. Furthermore, our results from the analysis of PAH model clearly showed that there was a correlation between death receptor signaling mediated by caspase -3/-8/-9 and ER stress. Moreover, the hypoxia-induced up-regulation of ER stress was in tandem with Nox4 induction (Figure 5A), which prompted us to examine the specific mechanisms regulating Nox4 signaling. In both cases, attenuated ER stress resulted in a significant reduction in Nox4 expression and MFI of ER tracker staining (Figure 5C). Taken together, these studies outline the critical role that anti-oxidative effect of H_2_S inhibits ER stress via Nox4 pathway in PAH (Figure 6).

**Figure 6:** Schematic diagram of the mechanisms of H2S in regulation of ROS and Nox4 in PASMCs Nox4 exhibit distinct subcellular locations in PASMCs from hypoxia-induced PAH rats. Of note, exogenous H_2_S inhibits ER stress via suppressing the NADPH activity and ER stress is able to be blocked by decreasing in Nox- expression and activity after interfering by H_2_S.

In the present study, we focus on the PASMCs and do not address potential direct effects of H_2_S on PA endothelial cells, which also contribute to plexiform lesions and vascular remodeling in PAH patients. Recent work has suggested that human PAH–PA endothelial cells are proliferative and share a very similar mitochondrial suppression with PAH-PASMCs; thus we speculate that a similar mechanisms could be involved, but more studies need further investigation. In addition, our studies did not directly address the potential effects of H_2_S on the right ventricle. However, GYY4137-treated animals had improved CO and performance on the treadmill test, consistent with improved cardiac function.

Although ER stress has not been definitively linked with all known triggers of PAH, this work, along with our recently published work, strengthens the evolving metabolic theory of H_2_S and links two fundamental cellular processes, ER stress and mitochondrial biology, potentially opening new avenues for therapies in diabetes cardiomyopathy and PAH [11,31]. Overall, genetically targeting ER stress for PAH prevention/therapy may be difficult to achieve. There are many proteins involved in this pathway and timing/threshold levels are of key importance to reverse PAH remodeling. Furthermore, this duality in survival vs. death results in tissue specific changes that are difficult to study in animal models with a total knockout of ER stress proteins or Nox4. As a result, an inducible and tissue-specific Nox4 KO system could be a potentially better *in vivo* model for future studies. For our experiments, GYY4137 inhibition of ER stress *in vivo* proved to be a more useful approach than the genetic inhibition.

## Availability of Supporting Data

We declare that materials described in the manuscript, including all relevant raw data, will be freely available to any scientist wishing to use them for non-commercial purposes, without breaching participant confidentiality.

## Availability of Data and Materials

The datasets used and/or analyzed during the current study are available from the corresponding author on reasonable request.

## Abbreviations

CAT: catalase
CCK-8: cell counting kit-8
CHOP: C/EBP-homologous protein
CO: cardiac output
CSE: cystathionine γ-lyase
DCF: 2′,7′-dichlorofluorescein
DCFH-DA: 2,7-dichlorofluorescein diacetate
EdU: 5-Ethynyl-2′-deoxyuridine
ER: endoplasmic reticulum
FBS: fetal bovine serum
H_2_S: hydrogen sulfide
MFI: mean fluorescence intensity
MPTP: mitochondrial permeablity transition pore
NAC: N-acetyl-l-cysteine
NOX4: NADPH oxidase 4
PAH: pulmonary arterial hypertension
PASMC: pulmonary artery smooth muscle cell
ROS: reactive oxygen species
SOD: superoxide dismutase
SR: sarcoplasmic reticulum
STZ: streptozotocin
